RETRACTED

# Preserving the Privacy of Healthcare Data over Social Networks Using Machine Learning

**DOI:** 10.1155/2022/4690936

**Published:** 2022-05-05

**Authors:** T. Veeramakali, A. Shobanadevi, Nihar Ranjan Nayak, Sumit Kumar, Sunita Singhal, Manoharan Subramanian

**Affiliations:** ^1^Department of Data Science and Business Systems, School of Computing, SRM Institute of Science and Technology, Kattankulathur, Chennai, India; ^2^Sri Venkateswara College of Engineering Technology, Chittoor, India; ^3^Indian Institute of Management, Kozhikode, India; ^4^Department of Computer Science and Engineering, Manipal University Jaipur, Jaipur 303007, India; ^5^Department of Computer Science, School of Informatics and Electrical Engineering, Hachalu Hundesa Campus, Ambo University, Ambo, Ethiopia

## Abstract

A key challenge in clinical recommendation systems is the problem of aberrant patient profiles in social networks. As a result of a person's abnormal profile, numerous vests might be used to make fake remarks about them, cyber bullying, or cyber-attacks. Many clinical researchers have done extensive study on this topic. The most recent studies on this topic are summarized, and an overarching framework is provided. When it comes to the methods and datasets that make up the data collection, the feature presentation and algorithm selection layers provide an overview of the various types of algorithm selections available. The categorization and evaluation of diseases and disorders has been one of the major advantages of machine learning in medical. Because it was harder to predict, it rendered it more controllable. It might range from difficult-to-find cancers in the early stages to certain other illnesses spread through the bloodstream. In healthcare, we may pick methods in machine learning depending on reliable outcomes. To do so, we must run the findings through each method. The major issue arises during information training and validation. Because the dataset is so large, eliminating mistakes might be difficult. The providers, other characteristics, various algorithms, data labelling techniques, and assessment criteria are all presented and contrasted in depth. Detecting anomalous users in medical social networks, on the other hand, is a work in progress. The result evaluation layer provides an explanation of how to evaluate and mark up the results of the various algorithm selection layers. Finally, it looks forward to more study in this area.

## 1. Introduction

With the widespread application of the development of mobile Internet technology, online healthcare social networks have quickly become an essential part of people's network life due to their convenience, flexibility, and rich content. However, the vast user privacy information in healthcare social networks and its vast commercial value have often become the targets of criminals who attempt to commit illegal activities. Among them, abnormal users are one of the standard methods criminals use to attack healthcare social networks. For example, merchants distort product value orientation for commercial interests [1–3]; criminals use multiple vests to deceive Internet users, steal information, or even online fraud [4–6]. According to statistics, the types of abnormal users also show a variety of forms due to different types of healthcare social networks. As shown in Table 1, they are widely present on different social platforms. For example, as of June 2012, Face book has about 8.7% (8.3 × 107) fake users, while Twitter faces the same problem. About 5% of users are fake users. Some experts believe that this proportion is possible up to 10% [7].

RETRACTED

Abnormal users in healthcare social networks have a wide range of existence and severe harm. Related scholars have summarized the research on the detection technology of strange users in healthcare social networks. Sun et al. [8] summarized the status quo and associated technologies of abnormal patient profile and abnormal behaviour detection in healthcare social networks. Song et al. [9] focused on analysing malicious patient profile algorithms and their applications based on features, space, and density. In the study by Hu et al. [10], focusing on four aspects of traditional spam, false comments, spam, and link factories, network characteristics, content characteristics, and behaviour characteristics are extracted. It explains the application of clustering algorithms, classification algorithms, and graph algorithms. For the problem of false information detection, Yuan et al. [11] studied graph-based algorithms. They divided them into subgraph analysis and mining algorithms, label transfer algorithms, and hidden factor decomposition algorithms. The research mentioned above only summarizes the current work from features or algorithms and is not comprehensive enough.

This article summarizes the implementation process of social network abnormal patient profile technology, as shown in Figure 1. The data collection layer introduces data acquisition methods and related data sets; the feature presentation layer explains attributes features, content features, network features, activity features, and additional features; the algorithm selection layer introduces supervised, unsupervised, and graph algorithms; the result evaluation layer explains data labelling methods and method evaluation indicators.

This research is organized as follows.  Section 1 describes the introduction, the supervised algorithm is described in Section 2, Section 3 describes the unsupervised learning, the graph algorithm is described in Section 4, Section 5 describes comparison of different algorithms, evaluation parameter is described in Section 6, and finally Section 7 describes the conclusion part.

RETRACTED

## 2. Supervised Algorithm

When the acquired data contain tags, the researchers design numerical features based on the idea of classification and divide users into abnormal users and regular users to detect strange users. Supervised algorithms can be divided into single classification algorithms and integrated classification algorithms:

1. Single classification algorithm refers to using only one classification algorithm to detect abnormal users. Commonly used is logistic regression, support vector machines, decision trees, and so on. Tara [5] and Qi et al. [7] used logistic regression to detect malicious users in Twitter and phishers in CNN and found that the name language pattern feature is the most significant feature that distinguishes malicious users from normal users. Jiang et al. [12] used logistic regression to detect false reviews in Amazon. According to the classification of products and assessments, it emphasizes detecting 4 more dangerous faulty comment areas. It is found that the characteristics of response activities are the most effective for the problem, and Zhu [2] found that the overall score deviation is essential for detection. Fake comments have no effect. Meng et al. [13] used support vector machines to detect Wikipedia's vests and found the 30 features that contributed the most to the problem through experiments. Zhang et al. [14] used support vector machines to detect abnormal behaviors of network users. Tables 2 and 3 show the comparison of detection characteristics and classification of detection algorithm, respectively.
2. The spammers in Twitter introduce the parameter *J* into the support vector machine to give the prior distribution of spammers, adjust *J* to balance the improvement in accuracy or recall, and select through gain and chi-square tests. There are several distinguishing characteristics. For example, Venkatesan et al. [15] used decision trees to detect cultural attackers in Wikipedia, sacrificed part of the accuracy requirements to achieve a higher recall rate, and won the 2010 PAN competition. Wang et al. [16] used decision trees and Bayesian network algorithms to detect false news about Hurricane Sandy on Twitter and found that the effect of decision trees is better. In addition, the contribution of text features is relatively significant. When transaction data (super clever agreement) technique is combined with traditional relational database strategies, data security, authenticity, time management, and other aspects of data regime are significantly improved. Logistic regression was employed by Jiang et al. [12] to detect fake reviews on Amazon. It stresses on four more risky defective remark areas, according with categorization of items and evaluations.
3. Integrated classification algorithm integrates multiple single classification algorithms to obtain higher accuracy, such as random forest, Adaboost, etc. For example, Kanhere et al. [17] used the random forest algorithm to detect abnormal users in discussion communities such as CNN. They found that the longer the sample time, the worse the prediction accuracy of the method, which confirmed that changes in user behaviour quickly lead to abnormal users. Wang et al. [18] used six classification algorithms, including random forest and Bayesian network, to detect the vests in Wikipedia. They found that the best features were reply frequency, increased bytes, and average contribution through experiments. Noh et al. [19] used the Adaboost method which detects the political navy in Twitter, uses the chi-square test to give the 10 most contributing characteristics, and analyzes the characteristics of the discovered political navy. Shalash et al. [20] used support vector machines, random forests, and Adaboost methods to detect deception in healthcare social networks. The Adaboost way is more effective, and this newly defined indicator is more effective. Bhanumurthy et al. [21] integrated Bayesian, NSNB, Winnow, and other algorithms into linear joint algorithms and obtained the effectiveness of each algorithm for the problem by optimizing the weights.

RETRACTED

## 3. Unsupervised Algorithm

When the sample data do not contain labels or contains few titles, based on the idea of clustering, researchers propose to use unsupervised learning algorithms to solve the problem of abnormal patient profile. Unsupervised algorithms are divided into decomposition mining from top to bottom and cluster mining from bottom to top.

1. *Decomposition Mining Algorithm from Top to Bottom*. When there is no label for the sample data, the researchers detect abnormal user groups by decomposing the social network graph. Perez et al. [22] constructed an SVN network based on topic similarity, deleted a part of edges based on text feature similarity to form an SPN network, clustered and mined abnormal users' group communities based on the similarity of modulus, and gave the accuracy of the method. The TIA algorithm [23] initializes normal users and malicious users according to different centrality value boundaries, then takes various decomposition diagram operations according to different attack modes, and continuously updates malicious users and regular user groups to achieve the purpose of predicting malicious users in the Slashdot network. The D-CUBE method [24] decomposes the relationship tensor by deleting the attribute value dimension with the largest cardinality or density, until an abnormal group is left at the end, and iteratively obtains multiple deviant user groups. This method uses a distributed algorithm. It is suitable for large-scale graph data format. The ND-SYNC method [25] is directly based on the RTFRAUD way for community discovery of the constructed feature space, using the deviation of internal and external synchronization to detect group anomalies and find Fake users in Twitter. There are various attributes of the data set to decide the user is abnormal or normal such as labelling method. In order to evaluate aberrant user detection systems, you must first learn how to label data. The labelling results are not persuasive despite the fact that his characteristics are simple and easy to implement; however, the data base has a high accuracy rate. It is difficult to control from the web page.
2. *Bottom-Up Cluster Mining Algorithm*. When a part of the data sample labels are available, the researchers use the similarity and known label samples to cluster the graph structure to solve the problem of abnormal user group detection. The Copy Catch method [26] mainly constructs the time matrix of healthcare social networks, clusters to maximize the number of strange users in the core of TNBC, detects abnormal user attack groups in Face book, and provides proof of stability and convergence. He et al. [27] constructed similar groups based on the MD5 similarity of the text and the same clustering of the URL pointing to the target and then judged whether each group is a fake user group through the distribution coverage of counterfeit users and the time burst. Lin et al. [28] found a method called Eigen–Spoke's new model and used the model's score to cluster samples until the model no longer increased to detect the social network and user groups. Jain et al. [29] initialized a small number of robots in Twitter and clustered them using the similarity of text information until a sufficient number of robots were found. The Catch-Sync method [30] redefines synchronization and normality.

RETRACTED

## 4. Graph Algorithm

Graph algorithms are becoming increasingly popular for spotting unusual users due to the increasing importance of network architecture and activity factors found in graph data. Among graph-based algorithms, spectral decomposition and random walks are two of the most commonly used techniques.

According to this approach, processing results in a characteristic matrix may be corrupted in order to create alternative groups. Scholars have worked hard to use spectrum-based decomposition methods to solve the problem of patients with aberrant profiles. If you look at [25], for example, the author created a hierarchical tree structure, combined the content matrix with a sparse representation, and then utilised the spectral decomposition simulation approach to iterate the optimal weights in order to discover the deceiver further. According to [29], the author used both a content matrix and a random walk network matrix to get the final result. Spammers on Twitter were tracked down using the spectral decomposition approach. Following [31], a new method was devised by author that integrated emotional information into both content and adjacency matrixes. However, there have been contributions from other researchers. As an example, author in [32] used a threshold and a seed to generate a kid.

Using the subgraph, the figure decomposes it into a smaller subspace in order to determine whether or not the user in the subspace is a phony YouTube user. The FEMA method [33] decomposes the three-dimensional tensor at different times to get the mapping matrix and the core tensor according to specified regularization criteria in response to the growth in the dimension of impact, notably the time component. It also increases your chances of being a strange user. To better identify assaults, the author in [17] employed SVD matrix decomposition to rebuild the degree of network nodes and imposed a restriction on the degree to better hide them from detection.

In the random walk algorithm, the node transition path is calculated, the unknown node's relationship to the known node or the transition probability is determined, and if the unknown node is abnormal, it is determined. Currently, the system is used to identify vest accounts in healthcare social networks. Bhanumurthy and Anne [33] technique employs a modified random walk algorithm to compute the transfer path of the node. If the node path and the path of the standard node cross, it is determined to be a regular user. However, each assault path may sustain at most *O* (*n* log *n*) vests node. If the end edge of the node path and the last edge of the standard node path coincide, then the user is considered a normal user and the number of tolerated vest nodes is reduced to *O* (log *n*) for each attack path [34]. The two approaches described above, however, can only identify one node as being inefficient in each cycle. This is how the author of [35] identifies multiple vest accounts quickly by taking random walks from a normal node and then performing a similar operation on a node, using the same bar to determine whether it is a vest or not. Then, using the discovered vest node and the same principle to identify multiple vest accounts, the author can quickly identify multiple vest accounts. Assigning credibility levels to other nodes using the Sybil Rank algorithm [4] involves using the random walk algorithm. According to the standardized and degree value findings, the nodes with a lower credibility value are placed at the bottom of the list. It is a suspicious node. Markov random fields are used in the Sybil Belief approach [13] for detecting vesting accounts. To begin, a random value is assigned to each node in the network to determine if it is a normal or vest node. Then, using a Markov random field, each node's posterior probability is determined. To put it another way, there is a 50% chance that the node is not abnormal.

RETRACTED

## 5. Comparison of Different Algorithms

Various detection algorithms have their advantages and disadvantages and have their application scenarios, as shown in Table 4, which lists the advantages and disadvantages of different detection algorithms.

### 5.1. Method Evaluation Layer

After selecting the appropriate feature representation and algorithm selection, researchers need to evaluate the effect of the method to a certain extent and need to obtain data annotations and method evaluation indicators.

### 5.2. Data Labelling Method

How to label data is a prerequisite for evaluating abnormal user detection methods. Although his features are simple and easy to implement, the labelling results are not convincing; however, the blacklist has a high accuracy rate. It is not easy to manage from the website.

## 6. Evaluation Parameter

Generally, the commonly used method evaluation indicators include accuracy, recall, precision, F1-score, and ROC (AUC) curve index. The researchers propose using unsupervised learning methods to overcome the problem of anomalous patient profiles when the sample data do not have labels as few titles, based on the principle of clustering. The finding analysis layer explains how to assess and mark up the outcomes of the several methods selection stages. The ROC curve is a curve drawn based on the confusion matrix's actual rate and false positive rate values as the coordinate axes, and AUC represents the area under the ROC curve. These indicators are based on a confusion matrix, and the definitions of various indicators are shown in Table 5.

This paper presents comparative analysis over supervised machine learning (SVM) and graph technique to identify abnormal patient profiles for reliable healthcare data over two healthcare dataset, i.e., Pubmed [36] and Medhelp [37]. It determines that the SVM leads over graph-based technique (GBT) and acquires 89%–92% accuracy, whereas SVM gains only 81%–84% accuracy over Pubmed (PM) and Medhelp (MH) dataset, respectively, as shown in Table 6 and Figure 2.

RETRACTED

However, SVM gains 78.28%–81.86% and GBT acquires 74.12%–76.52 precision over Pubmed (PM) and Medhelp (MH) dataset, respectively, as shown in Table 6 and Figure 3.

However, SVM gains 65.64%–69.84% and GBT acquires 75.52%–76.52% recall over Pubmed (PM) and Medhelp (MH) dataset, respectively, as shown in Table 6 and Figure 4.

However, whereas SVM gains 75.52%–76.24% and GBT acquires 86.61%–88.34% F1-score over Pubmed (PM) and Medhelp (MH) dataset, respectively, as shown in Table 6 and Figure 5.

## 7. Conclusion

With the gradual increase in the influence of healthcare social networks, more and more malicious users are focusing their attacks on healthcare social networks. Among them, the harm of abnormal users to healthcare social networks seriously threatens the information security of healthcare social networks and even the safety of users' property and life. To this end, in response to the problem of abnormal patient profile in healthcare social networks, this paper proposes an overall architecture. The processing architecture of the problem is explained separately from the data collection layer, feature representation layer, algorithm selection layer, and result evaluation layer and different data. The conclusion assessment layer explains how to assess and sign up the outcomes of the several algorithm selection stages. Finally, additional research in this area is anticipated. One of the future scopes of this research is that it will play a crucial role for comparing the effectiveness of supervised machine learning (SVM) and graph techniques for identifying aberrant patient profiles in two healthcare datasets. As the impact of healthcare social networks grows, more bad individuals are concentrating their attacks on them. Unusual users' harm to medical social networks is one of them, and it poses a severe threat to the data security of healthcare social networks, as well as the protection of users' property and lives. The sources, other features, different algorithms, different data labelling methods, and evaluation criteria are summarized and compared in detail. However, detecting abnormal users in healthcare social networks is an evolving process.

## Figures and Tables

**Figure 1:** Abnormal user architecture of healthcare social networks.

**Figure 2:** Accuracy of SVM and graph-based technique.

**Figure 3:** Precision of SVM and graph-based technique.

RETRACTED

**Figure 4:** Recall of SVM and graph-based technique.

**Figure 5:** F1-score of SVM and graph-based technique.

**Table 1:** Types of abnormal users.

Abnormal user types	Main existence platform
Spammer	Twitter, Weibo platform, CNN, Amazon, Yelp
Hoaxes	Wikipedia
Bot	Twitter
Sock-puppet	Wikipedia, Twitter, Facebook, CNN
Troll	Slashdot zoo, Wikipedia
Fake user	Google, Twitter, Amazon
Vandal	Twitter, Wikipedia, TCP

**Table 2:** Comparison of detection characteristics.

Detection feature	Features	The essential	Feature evaluation
Attribute characteristics	Using artificial design methods, it is easy to bypass attackers. The algorithm design is simple; the efficiency is low, the accuracy rate is relatively low, the data level is trim, and it has strict privacy protection.	Breakthrough privacy protection	Uncommonly used

Content characteristics	Natural language processing method is adopted, which is easy to be bypassed by attackers. In addition, the algorithm design is complicated, the efficiency is low, the accuracy rate is relatively low, the data level is significant, and the privacy protection is slight.	Design complex algorithms and reasonable language models	Commonly used

Network characteristics	Adopting complex network processing methods, not easy to be bypassed by attackers, simple algorithm design, low efficiency, relatively low accuracy rate, significant data level, and no privacy protection.	Master the global structure	Mainstream

Activity characteristics	Using behavioural pattern analysis and processing methods, it is not easy to bypass attackers; the algorithm design is simple, the efficiency is high, the accuracy rate is high, the data level is significant, and the privacy protection is slight.	Select the most distinguishable activity information	Mainstream

Auxiliary features	Using time-series model analysis, it is not easy to bypass attackers; the algorithm design is complex, the efficiency is high, the accuracy rate is high, the data level is trim, and it has slight privacy protection.	Effective use of time dimension information	Popular

**Table 3:** Classification of detection algorithms.

	Algorithm	Thought	Algorithm key issues
Supervised algorithm	Single classification algorithm	Classification	Select the key feature with the greatest degree of discrimination
	Integrated classification algorithm		

Unsupervised algorithm	Decomposition mining from top to bottom	Clustering	Choose a reasonable similarity index
	Cluster mining from bottom to top		

Graph algorithm	Spectral decomposition	Graph outlier detection	Processing large-scale sparse graph data
	Random walk		

**Table 4:** Comparison of detection algorithms.

Detection algorithm	Advantage	Shortcoming
Supervised algorithm	(1) High accuracy	(1) Need to include label data
	(2) Fast detection speed and high efficiency	(2) Need to train in advance
	(3) Mature algorithm design and mature deployment technology	(3) Need to select distinguishing features
	(4) Good real-time	(4) The selected features are easy to be bypassed by attackers, and the unknown mode detection effect is poor

Unsupervised algorithm	(1) Only need not contain label data	(1) Low accuracy
	(2) No need to train in advance	(2) The algorithm design is complicated, and the efficiency is low
	(3) Effective detection of unknown patterns	(3) Poor real-time performance

Graph algorithm	(1) Only graph data are needed	(1) Low accuracy and poor real-time performance
	(2) No need to train in advance	(2) The theoretical assumptions are complicated, and the reality is untenable
	(3) Effective detection of unknown patterns	(3) The algorithm design is complex, and the efficiency is low
		(4) There are different differences in social networks

RETRACTED

**Table 5:** Method evaluation indicators.

Methodological review Estimated index	Formal definition
Accuracy	*A*=TP+TN/TP+TN+FP+FN
Precision	*P*=TP/TP+FP
Recall	*R*=TP/TP+FN
F1-score	*F*=2*PR*/*P*+*R*
MCC	$\text{MCC}=\text{TP}*\text{TN}-\text{FP}*\text{FN}/\sqrt{\left(\text{TP}+\text{FP}\right)\left(\text{TP}+\text{FN}\right)\left(\text{TN}+\text{FN}\right)\left(\text{TN}+\text{FN}\right)}$

**Table 6:** Comparison of graph-based technique and SVM.

Technique	Accuracy		Precision		Recall		F1-score	
	PM	MH	PM	MH	PM	MH	PM	MH
Graph-based technique	81.56	84.24	74.12	76.52	65.64	69.84	75.52	76.24
SVM	89.32	92.14	78.28	81.86	75.52	76.52	86.61	88.34

## Data Availability

The data are available upon request.
